# Design and Simulation of Human Resource Allocation Model Based on Double-Cycle Neural Network

**DOI:** 10.1155/2021/7149631

**Published:** 2021-10-25

**Authors:** Qi Feng, Zixuan Feng, Xingren Su

**Affiliations:** ^1^Panzhihua University, Panzhihua 617000, Sichuan, China; ^2^Hongkong Shue Yan University, Hongkong 999077, China

## Abstract

The rationalization of human resource management is helpful for enterprises to efficiently train talents in the field, improve the management mode, and increase the overall resource utilization rate of enterprises. The current computational models applied in the field of human resources are usually based on statistical computation, which can no longer meet the processing needs of massive data and do not take into account the hidden characteristics of data, which can easily lead to the problem of information scarcity. The paper combines recurrent convolutional neural network and traditional human resource allocation algorithm and designs a double recurrent neural network job matching recommendation algorithm applicable to the human resource field, which can improve the traditional algorithm data training quality problem. In the experimental part of the algorithm, the arithmetic *F*1 value in the paper is 0.823, which is 20.1% and 7.4% higher than the other two algorithms, respectively, indicating that the algorithm can improve the hidden layer features of the data and then improve the training quality of the data and improve the job matching and recommendation accuracy.

## 1. Introduction

With the development of artificial intelligence technology, the intelligent process of enterprises is also advancing rapidly, which is reflected in two aspects of management intelligence and equipment automation [1]. As an important part of management intelligence, intelligent management of human resources is being paid more and more attention by more and more enterprise organizations [2, 3]. The rational management of human resources is of great help to enterprises in efficiently cultivating talents in the field of enterprises, perfecting the management mode of enterprises and improving the overall resource utilization rate of enterprises, which can effectively strengthen the integrity of enterprises and at the same time give better play to the economic and social value of enterprises [4]. Therefore, it is especially important to carry out efficient and intelligent human resource management for enterprises.

However, the distinctive feature of the intelligent era is the explosive growth of data, which makes the traditional human resource management methods no longer able to meet the massive data processing needs. The simple HR management system cannot make accurate analysis and deployment of the enterprise's manpower data and also wastes a lot of data collected by various information systems of the enterprise [5]. This not only loses the enterprise's information resources, but also slows down the intelligent information process. Therefore, it is necessary to apply advanced artificial intelligence algorithms to the enterprise human resource allocation system, which can significantly improve the processing capability of enterprise human resource data [6, 7].

Fundamentally, the processing of data is data mining. Data mining refers to the use of software systems to reasonably extract the useful information contained in the data, and most traditional data mining methods use statistical methods [8]. Statistical methods can be used in the case of small data content, but if there is a large amount of data, statistical methods are less able to adapt to the need. Machine learning is a widely used data mining method that can be trained on large amounts of data and extract the hidden features of the data [9]. These features are then continuously learned, and data information extraction can be performed accurately. In this paper, machine learning method is used to process human resource data and then improve the human resource data processing capability.

This paper focuses on the optimization of the composition of the human resources structure in terms of personnel categories, which is to accurately forecast the future human resources demand for each department and each type of position for the enterprise in advance, so as to improve the recruitment efficiency, avoid human resources shortage, and guide human resources training, thus maintaining the stable operation of the enterprise and preventing business risks [10]. Forecasting is the estimation and extrapolation of the future, which studies the future development of things and their operational rules and estimates and analyzes the trend of changes of its various elements. In order to achieve this purpose, it is often necessary to imitate or abstract the real world (object), and this process is called modeling; a representation and embodiment of the real world (object) obtained by means of modeling is called a model [11]. All objectively existing things and their movement forms are collectively called reality; reality and the future are not the same, but the future can be foreseen through the study of reality, which is prediction. From the perspective of information movement, reality contains the future and nurtures the future. Therefore, a “good” model should not only reflect reality but also accurately predict the future development. Thus, it is necessary to build a mathematical model that is in line with the objective development of things to make predictions.

Human resource demand recommendation is a human resource planning activity that takes the organization's established goals, development plans, and work tasks as the starting point and takes into account the influence of various internal and external factors to forecast the quantity, quality, and structure of human resources required by the organization in a certain period in the future [12, 13]. Unlike traditional mathematical modeling methods, neural networks have the ability to simulate part of human imaginative thinking and find out the characteristic relationship (mapping) between the input (influencing factors) and the output (human resource requirements) through learning and memory association of historical data. In the artificial neural network, the explanatory variables in the historical sample data can be used as the input units of the neural network, and the output units are obtained after the operation of the neural network implicit layer weights and activation functions [14]. The objective function is selected; i.e., the appropriate neural network weights are chosen to minimize the sum of squares of the difference between the desired output and the actual output of the neural network. Through multisample learning, the weights are modified and the deviation is continuously reduced so that the explanatory variables are optimally fitted to the explanatory variables, and the new known explanatory variables are input into the neural network and the predicted values are output through the implicit layer [15].

Since the human resource structure of an enterprise is a function of social, economic, political, and technological factors, modeling by conventional mathematical methods is not only a large workload but also difficult to guarantee accuracy [16]. Recurrent neural network has strong ability of nonlinear learning and pattern recognition, through which the relationship between human resource structure and its influencing factors can be modeled with relatively small error and high accuracy [17]. Neural networks have been used in a large number of applications in fiscal forecasting, management decision making, and process control. On the one hand, we can draw inspiration from the experience of neural network applications in other fields; on the other hand, we are required to design and develop new two-loop neural network models and algorithms in order to solve the problems of market research.

## 2. Human Resource Allocation Model Is Combined with Neural Network

### 2.1. Traditional Human Resource Allocation Model

According to the traditional human resource allocation theory, planning human resources mainly involves analyzing the personnel structure of the unit and sorting out the correlation between job requirements and personnel competencies in detail. Personnel competencies include various elements, which are weighted and summed to determine the quality score of personnel [18, 19].

The traditional HR scoring process is shown in Figure 1. First, the incoming data are grouped and analyzed into two groups: the personnel evaluation matrix and the personnel competency matrix [20]. The most commonly used is the employee competency matrix, which may take into account various factors, such as self-evaluation, superior-subordinate evaluation, and patient evaluation. The personnel competency matrix includes information such as employee performance, attendance, and job title. After obtaining the personnel evaluation matrix values and the personnel competency matrix values, the key indicator job match can be obtained as follows:where *n*_1_ ~ *n*_4_ is the corresponding evaluation parameter.


(1) $$\begin{array}{c} {\left(H_{ij}\right)}_{p\times q}=\left(n_{1}{\left(a_{ij}\right)}_{p\times 1}+n_{2}{\left(b_{ij}\right)}_{p\times 1}+\cdots +n_{4}{\left(d_{ij}\right)}_{p\times 1}\right). \end{array}$$

Let the other variable be *x*_*ij*_, with

(2) $$\begin{array}{c} x_{ij}=\left\{\begin{array}{cc} 1, & \text{assign personnel to corresponding positions,}\\ 0, & \text{not assigned to corresponding positions.} \end{array}\right) \end{array}$$

Therefore, the personnel can be optimized by the job matching model, as shown in the following equation:

(3) $$\begin{array}{c} \max Z=\sum_{i=1}^{n}\sum_{j=1}^{m}s_{ij}X_{ij},\\ \sum_{i=1}^{n}X_{ij}=1,\;j=1,2,\ldots ,m,\\ \sum_{j=1}^{m}X_{ij}\leq 1,\;i=1,2,\ldots ,n. \end{array}$$

The above algorithm is simple and effective and allows for a better allocation of human resources, but this is only applicable when there is little manpower data. As the enterprise system increases, the manpower data also increase, and the problem becomes complicated. This method is inefficient in calculation and does not allow for better data mining and effective management of human resources.

### 2.2. Improved Recurrent Neural Network Model

From the above, we can see that the essence of HR scheduling model is to analyze HR data and calculate the job matching score. Then the scheduling of personnel is based on the job matching score, which can be abstracted as a recommendation model in essence. Recommendation models have been analyzed and validated in many fields, and the current mainstream recommendation models use recurrent neural networks as the data processing module [21].

The most important feature of recurrent neural networks is the use of recurrent convolution for data training operations [22, 23]. The convolutional recurrent network model can be regarded as a hierarchical data model, and the input of the convolutional network is the original human resource data. Abstract features between the data are extracted through the process of recurrent convolution operation, pooling, and activation function, and the process is expressed as follows:

(4) $$\begin{array}{c} x^{1}⟶\omega^{1}⟶x^{2}⟶\cdots ⟶x^{L-1}⟶\omega^{L-1}⟶x^{L}⟶\omega^{L}⟶z,\\ z=f\left(x^{L},y\right). \end{array}$$

In this paper, *x*^*L*^ is the data input of *L* layer, *ω* is the parameter weight value of *L* layer, *z* is the loss function selected by the model, *y* is the calibration value of the model, and the function *f* is the final calculation parameter of the model. In this paper, the basic neural network is improved by using a hybrid recurrent neural network model, and the global model is combined with the local model to process the data by using the data features of the hierarchical model as the network output. The hierarchical model structure is then used to build the network and realize the job matching recommendation [24, 25]. The hybrid recurrent network model is shown in Figure 2.

In the process of model building, cross entropy [26] is selected as the loss functions in the paper. This loss function can compare the actual value of the data with the expected value of the data and then determine the closeness of the data, and the loss function is as follows:

(5) $$\begin{array}{c} L=-\sum_{n}\left(y\;\log\;p+\left(1-y\right)\log\left(1-p\right)\right). \end{array}$$

At the same time, the parameters are optimized during training using a gradient optimization algorithm. This way the parameter transfer can be as accurate as possible, and the specific update process of the model parameters is the following:

(1) The learning rate and the number of iterations of the neural network are updated as shown in the following equation:
  (6) $$\begin{array}{c} m_{t}=\beta_{1}m_{t-1}+\left(1-\beta_{1}\right)g_{t},\\ v_{t}=\beta_{2}v_{t-1}+\left(1-\beta_{2}\right)g_{t}, \end{array}$$
where *β*_1_, *β*_2_ are the hypermastigote of the recurrent neural network, *g*_*t*_ is the computational gradient of the model, and *t* is the number of iterations of the model.
(2) Optimal orientation of the first-order and second-order estimates [27] is
  (7) $$\begin{array}{c} {\hat{m}}_{t}=\frac{m_{t}}{1-\beta_{1}^{t}},\\ {\hat{v}}_{t}=\frac{v_{t}}{1-\beta_{2}^{t}}. \end{array}$$
(3) Update the parameters of the model from the results obtained above:
  (8) $$\begin{array}{c} \theta_{t+1}=\theta_{t}-\frac{l{\hat{m}}_{t}}{\sqrt{{\hat{v}}_{t}}+\varepsilon }. \end{array}$$

## 3. Algorithm Flow

As mentioned in Section 2.2, the overall algorithm used is the job matching recommendation algorithm. The process design of the recommendation algorithm should also be tailored to different application scenarios and data characteristics. Currently used algorithms in the HR field are usually statistical algorithms that do not take into account the hidden features of the data and rely on simple scoring and expert judgment mechanisms, which can easily lead to information scarcity problems [28].

In this paper, we combine recurrent CNN and traditional human resource allocation algorithm to design a job matching recommendation algorithm for human resource field. The algorithm not only improves the problem of low data training quality of traditional algorithms, but also effectively improves the data computation efficiency by using recurrent neural networks [29]. The core idea of the algorithm is to first extract the original features from the data, which are consistent with the features required by traditional human resources, including the personnel evaluation matrix and the personnel's ability matrix. The data are extracted and encoded in an encoder, and the encoded features are then fed as data input to the data input layer of RNN. The data are processed using the recurrent convolutional layer to obtain the job matching results, and the algorithm flow is shown in Figure 3.

First, the data is collected and selected using a distributed streaming collection method and grouped into a personnel evaluation matrix and a personnel competency matrix. The data are then abstracted, preprocessed, encoded using an encoder and saved to a data warehouse and further enhanced using a feature enhancement algorithm and fed into a RNN. The final job matching score is output and the HR recommendation process is completed.

The steps in the algorithm flow are described as follows:

1. Data collection: using the distributed streaming data collection method, the format of manpower data varies from company to company. Therefore, manpower data must be processed in a uniform format, including data rounding and conversion operations.
2. Preprocessing of the raw data: the datum is grouped so that a more comprehensive understanding of the HR model characteristics can be obtained. The datum is also saved to the data warehouse so that subsequent data model training can be supported.
3. Perform feature enhancement: the datum is obtained from the data warehouse and the results of data grouping are learned. Fused data results are used as neural network data input for network training.
4. Recommendation result output: the job matching results are ranked, and then the reasonable job assignment is made with reference to the score.

### 3.1. Algorithm Evaluation Metrics

The algorithms are evaluated by a certain number of metrics, and the accurate evaluation metrics are used in the evaluation of human resource recommendation algorithms in this paper [13, 22].

In the evaluation system, the higher the accuracy and recall, the better the algorithm. However, in some scenarios, accuracy and recall may be contradictory, so in order to synthesize these two metrics, the *F*1 value [30] is used in the paper for synthesis, and the formula is

(9) $$\begin{array}{c} \text{precision}=\frac{\text{tr}}{\text{tr}+\text{fr}},\\ \text{recall}=\frac{\text{tr}}{\text{tr}+\text{fnr}},\\ F1=\frac{2\cdot \text{precision}\cdot \text{recall }}{\text{precision}+\text{recall}}. \end{array}$$

## 4. Experiment and Analysis

### 4.1. Experimental Data

#### 4.1.1. Data 1

The data in this paper are sorted into three types of enterprise human resource data, including personnel information, personnel evaluation matrix values, and personnel capability matrix values. The datum was collected from 4,560 employees and 1,233 positions, with a sample size of 134,540 [31].

#### 4.1.2. Data 2

We included a large power supply company in a certain region; the details of the company are as follows: company A is the main power supply and management unit in the region, and the power supply covers 29 towns and 2 forest farms under the jurisdiction of the region, with a total of 31 secondary power supply companies; the company has been established for more than 30 years, and after a long period of development, the company's staff structure and business scope (service area) and quantity (mainly electricity sales and equipment) have changed dramatically. By 2020, more than 97% of the company's existing substations will be unmanned, and the service will be based on a network of eight 500 kV substations. With the deepening of market-oriented reform of the national power grid, the development of the company is facing new challenges, with management methods needing improvement, personnel structure needing optimization, and power supply equipment and facilities needing further upgrading. In this context, Company A has put forward the human resources slogan of “positive change, talent first” and strives to build a human resources management system to adapt to the new situation, striving to become a first-class power supply company in China and a leading player in the industry. Information on the company's human resources and company performance is mainly summarized through the company's information release [32].

Figure 4 depicts the trends of the number of employees and electricity sales of company A from 2010 to 2020. It can be seen that the number of employees of company A has been maintaining a growth trend with a relatively slow growth rate; and the electricity sales of company A, except for a certain downward trend around 2015, have generally maintained a good growth and still maintained a good growth in the recent year of total growth, for the decline in electricity demand during 2015 may be caused by factors such as the weakness of the domestic economy.

Although the number of employees of the company has maintained growth, the adjustment of relevant national policies and changes in the company's internal human resources structure have led to certain problems in the company's personnel structure, which is manifested in the high demand for power dispatching and transmission and substation personnel in the main power transmission network. In this regard, it is necessary for the company to plan its human resources department in advance, complete the human resources demand forecast as early as possible, adjust and optimize the personnel structure, clean up the surplus personnel, and introduce the insufficient number of professionals to serve the company's long-term development goals.

Through the above basic situation, it can be seen that the information related to the development history of company A is relatively detailed and rich in data, and the collected data shows certain volatility, which is suitable for the analysis and prediction of its human resource demand by using double-loop neural network.

### 4.2. Data 1 Experimental Test and Analysis of Results

In this paper, the samples are divided into a training sample set and a test sample set. The pseudocode of the neural network testing procedure is given in Algorithm 1

Then the feasibility of the algorithm in the paper is compared with the experiments, using the algorithm in the paper, CNN, and the traditional statistical method for model training and experimental analysis, and the analysis evaluation indexes are accuracy, recall, and *F*1 value. The experimental results are shown in Table 1.

As can be seen from Table 1, the *F*1 value of the algorithm in the paper is significantly improved compared with the other two algorithms, and the traditional statistical method is the least effective. *F*1 value is 0.678 in the case of large amount of data, and the *F*1 value of common CNN is improved to 0.766; the best performance of the algorithm in the paper is 0.823. This indicates that the direct use of recurrent convolutional network does not really improve the training features of the data, while the method of using global network plus local network in the paper can effectively improve the hidden layer features of the data and then improve the data training quality and improve the matching degree and recommendation accuracy of the algorithm.

### 4.3. Model Analytical Indexes and Screening in Data 2 Experiments

In this paper, we established the analysis index system of enterprise A and screened all the indexes based on the gray correlation method to determine the final key analytical indexes of human resources demand.

Based on the above principles, the following analysis indexes were selected as the initial analysis system of HR demand forecast for company A. The specific sinks are shown in Table 2.

After the construction of the original demand forecasting analysis system, we need to screen the indicators that affect the human resource demand of company A, i.e., the key indicators. The screening method is the gray correlation analysis method of calculating the comprehensive correlation degree, and the analysis results are summarized in Table 3. The correlation between each indicator and human resources is calculated by the gray system modeling software, and the specific results are as follows:


(10) $$\begin{array}{c} \rho_{a_{1}}=0.7896,\\ \rho_{a_{2}}=0.6157,\\ \rho_{a_{3}}=0.6875,\\ \rho_{a_{4}}=0.5792,\\ \rho_{a_{5}}=0.5680,\\ \rho_{a_{6}}=0.6080. \end{array}$$

The higher the value of the correlation, the greater the influence on human resources demand. By ranking the above correlations, we can get *a*_1_, *a*_2_, *a*_3_, *a*_4_: four variables with relatively large values, i.e., the length of transmission network, the number of substations, the total number of customers, and the amount of feed-in tariffs, have a greater influence on the analysis of human resources demand, so the above four analysis indicators are selected as key indicators [33].

### 4.4. Data 2 Forecast

The implementation of the double-loop neural network model consists of two stages: first, the key index prediction values are input into model to obtain the final prediction values.

The predicted values of key analytical indicators of human resource requirements of company A 2017–2019 are shown in Table 4.

Figure 5 shows the error trend of the neural network training. It can be seen that the output values obtained from the network training do not differ much from the optimal output values. The results are shown in Figure 6. *R* = 09999 is obtained, which initially indicates that our model is well trained.

The model was simulated using the historical data of 2019, and the actual output value of 6437 was obtained for 2019, and the relative error of its calculation was 1.067%, which was less than 3%. The data obtained from the GM (1, 1) model was used as the input of the neural network to predict the human resource demand of enterprise A from 2017 to 2019, and the relevant results are summarized as shown in Table 5.

According to the forecast results, enterprise A needs to further increase the total number of staff in T. The specific staffing requirements need to be adjusted according to the actual situation of the company.

### 4.5. Comparison of Different Models

In order to visually compare the prediction effects of different model, the prediction analysis of the two was carried out separately in this paper, and the specific results are shown in Table 6.

From the HR demand forecasting values of the two models in Table 6, it is clear that the forecasting results of the gray BP network forecasting model for each year are closer to the true values than the GM (1, 1) model [17, 34], which has better forecasting accuracy; meanwhile, the average relative error of the dual recurrent neural network forecasting model is only 0.1481%, which indicates that the model has very high forecasting accuracy. This indirectly indicates the applicability and reliability of the two-circulation neural network prediction model selected in this paper.

## 5. Conclusions

The essence of HR scheduling model is to analyze HR data and calculate the job matching score. Then the scheduling of personnel is performed based on the job matching score, which can be abstracted as a recommendation model in essence. In the paper, the basic neural network is improved by using a combination of a double-loop neural network model, a global model, and a local model, and the data features after the hierarchical operation of the model are used as the network output, and then the data is processed. By using a hierarchical model structure for network construction, we finally achieve high accuracy job matching and recommendation.

## Figures and Tables

**Figure 1:** HR scoring process.

**Figure 2:** Double-loop network model.

**Figure 3:** Algorithm flow.

**Figure 4:** Trend of the number of employees and electricity sales of company A from 2010 to 2020.

**Figure 5:** Prediction error results of our model.

**Figure 6:** Prediction results of our model.

**Algorithm 1:** : The neural network testing procedure.

**Table 1:** Comparative experimental result.

Model	Accuracy	Recall	*F*1
Model in this paper	0.8122	0.832	0.823
Statistical model	0.702	0.649	0.678
Cyclic neural network	0.755	0.775	0.766

**Table 2:** Company A's human resource demand forecasts analysis system.

Category 1 analysis index	Category 2 analysis indicators	Specific analysis indicators
Company development resources	Core resources owned by the company	Transmission network length *a*
		Number of substations under jurisdiction *a*

Market development of the company	Company market size	Total number of users *a*
		Total population served

Company development objectives	Company size	Annual revenue of the company
	Operating conditions of the company	Online electricity sales

**Table 3:** Summary of the results of the analysis of key indicators of human resources needs of enterprise A.

Particular year	Total number of users (10000)	Transmission network length (km)	Annual revenue of the company (million yuan)	Total number of employees (person)	Total population served (10000 households)	Online electricity sales (million kwh)	Number of substations under its jurisdiction (set)
2005	644.37	2018.57	8512.73	4718	145.63	28132.62	91
2006	644.52	2211.21	9753.721	4912	157.81	32143.82	97
2007	655.18	2501.24	10476.22	5098	162.97	36012.47	108
2008	669.75	2713.27	11678.13	5211	167.21	40231.92	119
2009	689.83	2851.42	13445.68	5423	171.23	44231.38	123
2010	693.18	3773.07	14621.95	5613	176.89	44315.27	134
2011	678.25	3385.29	15852.28	5662	186.24	42749.15	142
2012	681.31	3610.46	17246.77	5697	189.92	47531.83	151
2013	683.92	3910.79	20013.46	5907	202.43	49356.14	158
2014	690.71	4208.71	22143.92	6211	210.15	51897.15	162
2015	690.13	4427.43	24723.15	3248	218.32	53187.39	179
2016	690.56	4901.26	25923.84	6369	227.54	55582.17	190

**Table 4:** Predicted values of key indicators for the GM(1, 1) model.

Particular year	Total number of users (10000)	Number of substations under jurisdiction (station)	Transmission network length (km)	Online electricity sales (million kwh)
2017	248.13	206	5231.62	60003.17
2018	261.27	220	6243.99	62315.26
2019	270.52	233	6708.12	65103.82

**Table 5:** Summary of the prediction results of the trained BP network.

Particular year	2107	2018	2019
Predicted value (person)	6483	6549	6699

**Table 6:** Summary of the prediction results of the gray prediction model and our model.

Particular year	Actual personnel of the company (person)	Predicted value of GM model (person)	Predicted value of gray BP model (person)
2005	4718	4730	4723
2006	4912	4957	4956
2007	5098	5123	5109
2008	5211	5272	5262
2009	5423	5501	5472
2010	5613	5687	5632
2011	5662	5703	5682
2012	5697	5742	5715
2013	5907	5953	5928
2014	6211	6231	6220
2015	6248	6272	6261
2016	6369	6405	6264

Average relative error (%)	1.1154	0.1481	

## Data Availability

The dataset used in this paper is available from the corresponding author upon request.
